# A Novel Method for COVID-19 Detection Based on DCNNs and Hierarchical Structure

**DOI:** 10.1155/2022/2484435

**Published:** 2022-08-31

**Authors:** Yuqin Li, Ke Zhang, Weili Shi, Zhengang Jiang

**Affiliations:** ^1^School of Computer Science and Technology, Changchun University of Science and Technology, Changchun 130022, China; ^2^Zhongshan Institute of Changchun University of Science and Technology, Zhongshan, China

## Abstract

The worldwide outbreak of the new coronavirus disease (COVID-19) has been declared a pandemic by the World Health Organization (WHO). It has a devastating impact on daily life, public health, and global economy. Due to the highly infectiousness, it is urgent to early screening of suspected cases quickly and accurately. Chest X-ray medical image, as a diagnostic basis for COVID-19, arouses attention from medical engineering. However, due to small lesion difference and lack of training data, the accuracy of detection model is insufficient. In this work, a transfer learning strategy is introduced to hierarchical structure to enhance high-level features of deep convolutional neural networks. The proposed framework consisting of asymmetric pretrained DCNNs with attention networks integrates various information into a wider architecture to learn more discriminative and complementary features. Furthermore, a novel cross-entropy loss function with a penalty term weakens misclassification. Extensive experiments are implemented on the COVID-19 dataset. Compared with the state-of-the-arts, the effectiveness and high performance of the proposed method are demonstrated.

## 1. Introduction

The number of patients with the new coronavirus disease (COVID-19) has increased sharply, placing an unprecedented burden on the global systems. Especially in many countries, the healthcare systems have already been overwhelmed [1]. As of July 13, 2022, the total number of COVID-19 infective cases worldwide is 557,035,533, including 6,368,340 deaths. Some COVID-19 virus particles images are illustrated in Figure 1, which are released by the National Institute of Allergy and Infectious Diseases (NIAID) and Rocky Mountain Laboratories (RML) [2]. The clinical manifestations of COVID-19 are more complicated and may include fever, cough, and severe headache. There are not enough fully effective vaccines available for prevention of COVID-19. In view of this, people are easily infected by the droplet of coronavirus. Therefore, early detection of COVID-19 is very important to isolate suspicious patients immediately and reduce the possibility of infection in a healthy population. In recent years, Reverse transcription polymerase chain reaction (RT-PCR) has been used as the main method for screening COVID-19 [2]. However, RT-PCR is time-consuming and error-prone [3]. Chest radiography imaging (X-ray) and computed tomography (CT) can also be applied for pneumonia diagnosis. Compared with CT and magnetic resonance Imaging (MRI), chest X-ray is a cheap, fast, and common clinical diagnosis method. In addition, chest X-ray images can provide patients with lower radiation doses. Therefore, chest X-ray images are chosen in our study to detect COVID-19. However, making an accurate and correct diagnosis from chest X-ray images requires expert experience and knowledge [4]. In the early stage of COVID-19, a ground class pattern can be seen in the marginal areas of pulmonary vessels edges, which may be difficult to confirm visually. Diffuse airspace opacities or asymmetric patches of COVID-19 have also been reported. In fact, the differences between various lesions are small in chest X-ray images. It is difficult to detect lung disease solely on the basis of shape or area. That is, the representations between target classes are too similar, and the differences between classes are not obvious. It is difficult to interpret these subtle abnormalities. This issue leads to lower accuracy of lesion detection. Besides, considering the large number of suspected cases and the limited number of trained radiologists, there is an urgent need for efficient and automatic methods to identify COVID-19 [5].

## 2. Related Works

Deep convolutional neural networks (DCNNs) have been proven to be superior to traditional machine learning approaches due to their outstanding ability of automatic abstract features extraction. Many deep leaning-based methods have been proposed to detect COVID-19 cases from X-ray images effectively [6–11]. In general, deep learning-based methods require abundant labeled data. However, one of the most serious challenges in medical image analysis is the lack of available datasets. Furthermore, labeling a large amount of data by radiologists is time-consuming and costly. To conquer this dilemma, the concept of transfer learning is proposed, where models trained in one domain can be reused in another related domain. In actual scenarios, transfer learning is conducted by a CNN model trained on a larger dataset (e.g., ImageNet). Hemdan et al. [11] used DenseNet and VGG19 to diagnose COVID-19 from X-ray images. Uçar and Korkmaz [12] introduced a model called COVIDiagnosis-Net, which fine-tuned SqueezeNet pretrained network with the Bayes optimization. Bargshady et al. [13] adopted CycleGAN for data augmentation and then used InceptionV3 to detect COVID-19. Sahinbas and Catak [14] used X-ray images to detect COVID-19 with the well-known pretrained deep CNNs such as VGG-16, VGG-19, ResNet, DenseNet, and InceptionV3, and the experimental results have proven that the pretrained VGG-16 can detect COVID-19 with the highest classification performance. Punn and Agarwal [15] used ResNet, InceptionV3, and Inception networks separately to detect COVID-19. Ahuja et al. [16] developed three-steps to detect COVID-19 in CT images. The first step conducted data augmentation, the second step used transfer learning pretrained models to perform classification task, and the last step was abnormality localization using deeper layers. Singh et al. [17] used truncated VGG16 to extract features from the input images and then employed the principle component analysis (PCA) method for feature selection. Afshar et al. [18] introduced the COVID-CAPS model, which is an alternative framework based on the capsule network. Sarker et al. [19] used Densenet-121 to effectively detect COVID-19 cases.

The above methods used transfer learning-based methods to detect COVID-19. In fact, in order to obtain richer and more high-level features, the network structure is usually designed to be deeper or wider. However, the continuous increase in depth of a single network may cause the loss of discriminative details in the intermediate layers. Although these details can be low-level features, they may be essential for abnormalities in X-ray images that are difficult to classify. These problems have become obstacles and bottlenecks in the development of DCNNs.

In view of this, many researchers try to expand the width of the network to extract more useful feature information. Based on this idea, Hou et al. [20] proposed a novel framework which combined two isomorphic DCNN models to extract more features. Hosseinzadeh [21] concatenated different features extracted from AlexNet, ResNet50, SqueezeNet, and VGG19 networks. Gayathri et al. [22] integrated Xception and InceptionResNetV2 pretrained models for feature extraction. However, the features extracted from these isomorphic or similar networks may be duplicated. Chen et al. [23] proposed a dual asymmetric network called DualCheXNet, which integrated the ResNet and DenseNet to learn more discriminative features adaptively. ResNet adds input features to the output through residual blocks. In contrast, the input channels are concatenated with its outputs in each dense block of DenseNet structure. According to these properties, the ResNet enables us to reuse early features while the DenseNet tries to explore new features. Hence, it can be concluded that the features extracted from ResNet and DenseNet are unique and different and may be complementary.

In traditional classification method, a two-step procedure including hand-craft feature extraction and classification is generally conducted. Inspired by the previous discussion, different from the traditional methods, we employ an end-to-end network which can predict COVID-19 directly from X-ray images. In our research, we use a hierarchical structure with two identical configurations to detect COVID-19 cases. In the rest of this paper, we use “feature extraction network” to represent these two identical configurations. The feature extraction network comprises two different DCNNs, and the subnetworks are pretrained on the ImageNet dataset. The feature extraction network contains ResNet-50 and DenseNet-201 DCNNs. Behind the pretrained models, some auxiliary layers are added to improve the classification performance. The following are the main contributions of this paper:

1. This work uses a hierarchical structure containing two configurations to detect COVID-19 in stages. That is, the samples are distinguished as “normal” or “pneumonia” in the first stage. If a case is classified as “pneumonia,” the second classifier will distinguish whether it is pneumonia caused by “COVID-19”
2. At each stage of the two classification tasks, two asymmetric pretrained networks containing ResNet-50 and DenseNet-201 are integrated to extract more discriminative and complementary features
3. Behind the pretrained subnetworks, the original classification layers are discarded. An attention mechanism called SE module and a GlobalAveragePooling operation are used to improve the performance of classification tasks. By concatenating the features from the above architecture, three fully connected layers are included, and dropout mechanism is added to the fully connected layer
4. Based on the traditional binary cross-entropy (CE) loss function, the proposed framework utilizes a novel loss function by adding a penalty term to the traditional cross-entropy, which introduces a difference between the predicted and the true label probability values. With this novel loss function, the generation of optimal model has been accelerated to a large extent

The rest of the research is organized as follows.  Section 3 presents the proposed method in detail.  Section 4 shows some experimental results and the related detail discussion. Finally, Section 5 concludes the whole work.

## 3. The Proposed Method

### 3.1. Hierarchical Structure

For classification tasks, there is a certain relationship among interclass. In general, in actual scenarios, classes are organized in a hierarchical structure, which can be regarded as a tree. In our research, we adopt a hierarchical classification framework. We take the input as the root node, which is the target to be classified. The target classes are located in the leaves of the tree, and each parent node in the tree represents a classifier. The diagram of this research is given as Figure 2. In our research, two classifiers are needed, and one is at the root node, used to distinguish between the normal and pneumonia; the other is on the second layer, dedicated to distinguishing between the COVID-19 and non-COVID-19. Therefore, this research divides the classification task into two stages. At the first stage, the instance is input to the first classifier. If the result is predicted as “normal,” the inference ends. Otherwise, it will be fed to the second classifier. Then the second classifier will distinguish whether it is pneumonia caused by “COVID-19.”

### 3.2. Problem Definition and Formulation

In this section, we present the problem definition and formulation of this paper. In a broad sense, transfer learning refers to a learning strategy that uses the knowledge gained in solving one problem *S* to solve another problem *T*. We define transfer learning in terms of domain and task. The domain *𝒟* is defined by a feature space *𝒳* and a probability distribution *P*(*X*) defined on *𝒳*. The task *𝒯* is defined by a label space *𝒴* and a prediction function *P*(*y* | *x*). Next, we define two sets, one contains source domain and task (*𝒟*_*s*_, *𝒯*_*s*_), and the other contains target domain and task (*𝒟*_*T*_, *𝒯*_*T*_), where *𝒟*_*s*_ ≠ *𝒟*_*T*__*s*_, *𝒯*_*s*_ ≠ *𝒯*_*T*_. The purpose of transfer learning is to use the knowledge gained in learning from *f*_*s*_ for the subsequent learning task *f*_*T*_.

The proposed method consists of two asymmetric pretrained DCNNs to construct a wider architecture. This paper formulated this process with the formal definition putted forward in [23]. We define the input images of two pretrained networks as **I**_**P**_ and **I**_**Q**_, respectively, where **I**_**P**_ = {*p*_1_, *p*_2_, ⋯, *p*_*N*_}, **I**_**Q**_ = {*q*_1_, *q*_2_, ⋯, *q*_*N*_}, and *N* denotes the number of training samples. Specifically, the input images of the two subnetworks are the same. The feature map outputs of the different DCNNs are represented as **f**_**P**_ = *α*(**I**_**P**_, *x*) and **f**_**Q**_ = *α*(**I**_**Q**_, *x*), respectively. These two different feature spaces can complement each other. We use **C**_**F**_ to represent the classification results of the classifier, and **C**_**F**_ can be formulated as Equation (1). In addition, we use **L**_**F**_ to denote the loss of the classifier, and **L**_**F**_ can be formulated as Equation (2).

(1) $$\begin{array}{c} C_{F}=\delta \left(f_{F}\right)=\delta \left(f_{P}⊕f_{Q}\right), \end{array}$$

(2) $$\begin{array}{c} L_{F}=\varphi \left(C_{F}\right), \end{array}$$

where *δ* is a activate function and *φ* is the loss function.

### 3.3. Feature Extraction Network

The block diagram of the proposed method is shown in Figure 3. The overall classification task can be divided into two modules: feature extraction module and classification module. In the feature extraction module, it has attracted widespread attention in enhancing DCNN with larger capacity. To achieve this goal, the network is usually designed to be deeper or wider. Different from traditional “deeper” DCNN networks, this paper designs a “wider” architecture to learn richer features. Compared with a single DCNN model, concatenating different DCNNs will integrate different information to create a more discriminative and comprehensive feature representation. In this work, two asymmetric networks are integrated into a “wider” architecture. The core idea of this “wider” architecture is to learn richer and complementary features by different DCNNs. ResNet [24] uses global average pooling instead of fully connected layers. Besides, shortcuts are added between layers, which can prevent distortion as the network gets deeper and more complex. DenseNet [25] provides a compact and thinner structure that can achieve good performance with fewer parameters. It is instantly favoured for many medical image diagnostic tasks. This paper employs these two asymmetric networks to extract more discriminative features.

In this work, we use a hierarchical structure to detect COVID-19, which contains two identical configurations. The overall architecture of the proposed method is shown in Figure 4. The feature extraction network integrates ResNet-50 and DenseNet-201 models, which have been pretrained on the ImageNet dataset. The architecture of ResNet-50 is illustrated in Figure 5, starting with a convolutional layer and ending with a fully connected layer.  Figure 6 shows the network framework of DenseNet-121, which is a similar framework of DenseNet-201. This network is composed of 4 dense blocks. The structure between two adjacent blocks is referred to as transition layers, which can be used to adjust the sizes of the feature maps through convolution and pooling operations.

In our research, the original classification layers at the end of the DCNNs are discarded, and the SE block and a GlobalAveragePooling operation are added behind the pretrained DCNNs. SE network improves the representation ability of the network by explicitly modelling the interdependence between feature channels. The structure of SE block is shown in Figure 7, consisting of squeeze and excitation operations. After pretraining, the extracted features from two subnetworks are concatenated directly to form new feature vectors. The upper part of Figure 4 is the stage of feature extraction using transfer learning.

### 3.4. Classifier

The lower part of Figure 4 is the classification stage. In this stage, the features extracted from different subnetworks are concatenated. Then the concatenated features are fed into the classifier to generate classification outputs. In general, a fully connected layer is the last and the most important layer for DCNNs. The function of these layers is similar to a multilayer perceptron. In this work, three fully connected layers are constructed into the classifier. In addition, dropout mechanism is added to the fully connected layer, which is used to avoid overfitting. The activation function of the first two layers is ReLU, and the last is Softmax. The following equations give the definition of these two activation functions.

(3) ReLUx=0,if x<0x,if x≥0,

(4) $$\begin{array}{c} \text{Softmax}\left(x_{i}\right)=\frac{e^{x_{i}}}{\sum_{y=1}^{m}e^{x_{y}}}. \end{array}$$

### 3.5. Training Strategy

To coordinate the two extractors to learn complementary features, the training strategy plays a vital role. In this paper, we adopt an improved cross-entropy cost function to minimize the distance between the true label and predict probabilities. The basic cross-entropy is defined as Equation (5). In this research, we add a penalty term which introduces the difference between the predicted and the true label probability values as Equation (6). The penalty term can be formulated as Equation (7). By this way, it can assist the network to increase its capacity to focus on misclassification.

(5) $$\begin{array}{c} \ell_{ce}=-\overset{N}{\underset{i=1}{\sum }}p_{i}\log q_{i}, \end{array}$$

(6) $$\begin{array}{c} \ell_{loss}=-\frac{1}{N}\overset{N}{\underset{i=1}{\sum }}\left(p_{i}\log q_{i}+\ell_{penalty}\right), \end{array}$$

(7) $$\begin{array}{c} \ell_{penalty}=p_{i}q_{i}-q_{i}, \end{array}$$

where *p*_*i*_ and *q*_*i*_ represent the true label and predicted probabilities for each image, respectively. From Equations (6) and (7), it is clear that if the sample is classified correctly, the penalty term is 0. This cost function will be minimized by using stochastic gradient descent (SGD) algorithm.

## 4. Experiments and Discussion

### 4.1. Dataset

In this paper, an open-access dataset called COVID-19 radiography database [28] is used to estimate the performance of the proposed method. This dataset is available on the website: https://www.kaggle.com/tawsifurrahman/covid19-radiography-database/. This dataset was created by a team of researchers from some universities and hospitals, which comprises 1200 COVID-19 cases, 1341 normal images, and 1345 viral pneumonia cases [9].  Figure 8 shows a few examples of chest X-ray images of three categories.

For our research purposes, our experiments are conducted on two binary classification datasets (Dataset-1 and Dataset-2) corresponding to the two classifiers.

In Dataset-1, the classifier only distinguishes the class between “normal” and “pneumonia.”

In Dataset-2, the samples related to the “normal” class are removed. This dataset consists of samples related to pneumonia and COVID-19 cases.

In this research, considering the performance of software and hardware devices and avoiding the problem of data imbalance, we adjusted the dataset appropriately. More specifically, in the Dataset-1, we have randomly chosen 500 normal (healthy person) samples and 1000 abnormal cases for training. The 1000 abnormal cases included 500 viral pneumonia cases and 500 pneumonias caused by COVID-19. Therefore, the proposed method performs classification tasks on “normal” and “pneumonia” on Dataset-1. If the case was classified as “pneumonia,” it would be sent to the second classifier. Next, in the Dataset-2, we use the above 1000 abnormal cases including 500 viral pneumonia cases and 500 COVID-19-positive samples from the COVID-19 radiography database to train the second classifier.

In order to validate the trained model, we randomly selected 300 samples from the remaining dataset. The 300 samples consisted of 100 normal and 200 pneumonia cases. And the 200 pneumonia cases comprised of 100 COVID-19 and 100 viral pneumonia cases.

### 4.2. Data Augmentation

In the tasks of image-based supervised learning, augmentation strategy was widely applied in natural images. Geometric transforms (or affine transforms) were most commonly used in the training process [29]. For medical images, specific structures such as lesions and tissues are relatively sensitive to some operations. Excessive enhancement will distort the actual distribution of the training data due to the introduction of too many outliers. Therefore, it is necessary to choose the appropriate enhancement methods carefully. The data augmentation strategies used in this research were rotation, horizontal, and vertical flip.

### 4.3. Implementation Details

In this paper, all images were resized to 224 × 224 pixel size in the Dataset-1 and Dataset-2. We used the “ImageDataGenerator” class from Keras in Python to augment the dataset. The data augmentation was used with rotation = 90°, vertical flip = true, and horizontal flip = true. This paper adopted a training strategy with a novel loss function proposed in this paper, with a learning rate of 0.0001. Besides, 80% of the samples in the training dataset were reserved for training, and the remaining 20% was for validating. In this research, the pretrained networks were trained from scratch without freezing layers, and these two networks were trained separately. By this way, two binary classification models were obtained. The first classifier only distinguished the class between “normal” and “pneumonia,” and the second can distinguish whether it is pneumonia caused by COVID-19. All of the training processes in experiments were conducted for 50 epochs, with a batch size of 20.

### 4.4. Indicators

There are several metrics which can be applied to evaluate the performance of classification tasks. The indicators used in this research were accuracy, sensitivity, *F*1-score, precision, and specificity, which were formulated as follows, respectively.

(8) $$\begin{array}{c} \text{Acc}=\frac{\text{True positive }\left(\text{TP}\right)+\text{True negative }\left(\text{TN}\right)}{\text{Total number of tested images}}, \end{array}$$

(9) $$\begin{array}{c} \text{Sensitivity}=\frac{\text{TP}}{\text{TP}+\text{False negative}\left(\text{FN}\right)}, \end{array}$$

(10) $$\begin{array}{c} \text{Specificity}=\frac{\text{TN}}{\text{TN}+\text{False positive }\left(\text{FP}\right)}, \end{array}$$

(11) $$\begin{array}{c} \text{Precision}=\frac{\text{TP}}{\text{TP}+\text{FP}}, \end{array}$$

(12) $$\begin{array}{c} F1‐\text{Score}=\frac{2\times \text{Precision}\times \text{Sensitive}}{\text{Precision}+\text{Sensitive}}. \end{array}$$

### 4.5. Results and Discussion

We conducted 2 binary classifications with hierarchical structure for COVID-19 detection. In the first stage, the target samples were distinguished as “normal” or “pneumonia.” To validate our trained model, we selected 300 samples, including 100 normal and 200 pneumonia cases. The 200 cases of pneumonia consisted of 100 COVID-19 and 100 viral pneumonia cases. In the second stage, the cases classified as “pneumonia” from the first stage continued to distinguish whether it is pneumonia caused by “COVID-19.” For evaluating the trained model, the above 100 abnormal cases were used to distinguish whether pneumonia was caused by “COVID-19.” Finally, as shown in Table 1, the obtained sensitivity, specificity, precision, *F*1-score, and accuracy values of the proposed method were 99.00%, 100%, 100%, 99.50%, and 99.67%, respectively.

### 4.6. Ablation Analysis

The hierarchical structure to detect the COVID-19 is adopted in this paper. This structure can be regarded as a tree, in which the target classes were located in the leaves of the tree. To prove the validity of the hierarchical structure, this paper conducted a comparative experiment, which only trained the proposed model once, and directly classified the results into three categories: normal, pneumonia, and COVID-19. In order to ensure the consistency of the data, this comparative experiment used the same data as that from Section 4.1, which is 500 normal (healthy person) samples, 500 viral pneumonia cases, and 500 COVID-19-positive samples. And we also used the same test data to evaluate the comparative experiment. The experimental configurations were the same as the proposed method. We reported the performance of the comparative experiment and the proposed method in Table 1. It can be noted from Table 1 that the proposed hierarchical structure achieved higher performance under different evaluation indicators.

To prove the effectiveness of the proposed dual asymmetric network, we compared the proposed framework with their corresponding baseline single networks, ResNet-50 and DenseNet-201. In these experiments, we also used a two-stage hierarchical structure for COVID-19 detection. The experimental configurations were the same as the proposed method. Next, we analysed the classification results of the single baseline network and the proposed network.  Figure 9 shows the training and validation accuracy and loss analyses of 3 methods in the first stage. In this stage, the models were trained to distinguish whether the sample was “normal” or “pneumonia.” Figure 10 shows the training and validation accuracy and loss analyses of 3 methods in the second stage. In this stage, the models were trained to distinguish whether the “pneumonia” cases from the first stage were caused by “COVID-19.” From Figures 9 and 10, it can be noted that there is a significant improvement of the proposed method in accuracy and loss values. The obtained sensitivity, specificity, precision, *F*1-score, and accuracy values are summarized in Table 2, and our method achieved higher performance against other single models. Besides, compared with the corresponding baseline single DCNNs, the proposed method requires more time and a larger memory for model training.

Next, we discussed the effectiveness of the proposed novel loss function. In the training process, this paper proposed a novel trained strategy which added a penalty term to the traditional cross-entropy loss function. To prove its effectiveness, this paper conducted comparative experiments by using traditional cross-entropy loss function. The analysis of training and validation accuracy on Dataset-1 over 50 epochs is illustrated in Figure 11, and the Dataset-2 is given in Figure 12.  Figure 13 shows the analysis of validation loss on Dataset-1 and Dataset-2. Each of the subfigure of Figures 11–13 included the performance of traditional cross-entropy loss function and our improved cross-entropy cost function. It showed that the validation accuracy of the proposed method is 100% in 12 epochs in the first stage, and the validation accuracy of the proposed method is 100% in 13 epochs in the second stage. The training and validation accuracy of the proposed method were higher than the traditional cross-entropy loss function on the whole. In addition, it can be seen that the validation loss convergence value of the traditional method was larger than the proposed method. From Figures 11–13, we can conclude that the novel loss function by adding penalty term can increase its capacity to focus on misclassification and accelerate the convergence speed of the model.

### 4.7. Comparison Analysis

To evaluate the effectiveness of the overall proposed network, we compared our method to some state-of-the-arts for COVID-19 detection. Chen et al. [30] fused the pretrained MobileNet and SE block to form a new network. Apostolopoulos et al. [31] trained the MobileNet v2 from scratch to extract the features for COVID-19 detection, which had been proven to achieve outstanding performance in related tasks. Gayathri et al. [22] integrated Xception and InceptionResNetV2 pretrained models for feature extraction. Then these features were concatenated to an autoencoder for reducing dimensionality. Bargshady et al. [13] adopted CycleGAN for data augmentation and then used InceptionV3 to detect COVID-19. Irfan et al. [32] proposed a hybrid deep neural network (HDNN) model, which is a mixture of two deep learning models (LSTM + CNN). Almalki et al. [33] introduced a novel model called CoVIRNet (COVID Inception-ResNet) for COVID-19 detection. Nguyen et al. [34] concatenated features extracted from three pretrained deep CNNs for microscopic image classification. The three pretrained networks were Inception-v3, ResNet152, and Inception-Resnet-v2. Chen et al. [23] proposed a dual asymmetric model, which is a complementary combination of ResNet50 and DenseNet-121 networks. Moreover, an iterative training strategy was designed for training.

Table 3 displays the results of different literatures conducted on the same dataset used in this paper. The performance of the result was measured by five indicators including sensitivity, specificity, precision, *F*1-score, and accuracy. From Table 3, it was clear that the proposed method obtained superior performance compared to other studies. The advantages of the proposed method can be summarized as follows:

1. Compared with single network models, the “wider” architecture built a multifeature description structure, which can extract more and richer features from the input images by different DCNNs
2. Compared with other “wider” models, our research adopted a hierarchical structure to complete the classification task in stages, which can effectively solve the problem of misclassification caused by too similar representation between different objects. This mechanism was conducive to image exploration and analysis of COVID-19
3. In addition, we also made other improvements in training strategy and in network. The improved loss function and other improvements can make the model focus on significant features representation of the input images

The limitation of the proposed method is that no more datasets are used for model validation. The proposed method in this paper should be tested with more different kinds of datasets.

## 5. Conclusions

In this paper, we develop a novel framework to detect COVID-19 cases based on DCNNs and hierarchical structure. Specifically, two asymmetric pretrained subnetworks are integrated to construct a wider architecture, which can learn more discriminative and complementary features. To improve the performance of the feature extraction network, an attention mechanism based on SE block is introduced in the network. Then, two tasks are trained with a novel loss function which combines the cross-entropy with a penalty term. To verify the effectiveness of the above modules, a series of ablation analyses are implemented to show the contribution of each module of the proposed method. To validate the high performance of the overall algorithm, some comparative experiments are carried out. The results show that the proposed method achieves higher performance with the accuracy for COVID-19 classification. In future work, we will further improve the applicability of the algorithm so that it can cope with multiple disease classifications in medical image analysis.

## Figures and Tables

**Figure 1:** Images of COVID-19 virus particles: (a) captured by scanning electron microscope; (b) captured by transmission electron microscope.

**Figure 2:** Hierarchical classification presentation. Each parent node in the tree represents a classifier, and each leaf node is a category.

**Figure 3:** The block diagram of the proposed method with transfer learning.

**Figure 4:** The architecture of the proposed method, in which the upper is transfer learning for feature extraction and the lower one is classifier.

**Figure 5:** Pretrained ResNet-50 network [26].

**Figure 6:** DenseNet-121 structure with four dense blocks and three transition layers [8].

**Figure 7:** The squeeze and excitation structure [27].

**Figure 8:** Some examples of chest X-ray images of three categories: normal (healthy person), viral pneumonia (patients suffering from viral pneumonia), and COVID-19 (pneumonia caused by COVID-19).

**Figure 9:** Training and validation analysis of the first stage over 50 epochs. (a, b) Comparisons of 3 different models. In this stage, the models were trained to distinguish whether the sample was “normal” or “pneumonia”.

**Figure 10:** Training and validation analysis of the second stage over 50 epochs. (a, b) Comparisons of 3 different models. In this stage, the models were trained to distinguish whether the “pneumonia” cases from the first stage were caused by “COVID-19”.

**Figure 11:** Training and validation accuracy analysis of the first stage on Dataset-1 over 50 epochs. (a, b) Comparisons of the traditional cross-entropy loss function with our improved cross-entropy cost function.

**Figure 12:** Training and validation accuracy analysis of the second stage on Dataset-2 over 50 epochs. (a, b) Comparisons of the traditional cross-entropy loss function with our improved cross-entropy cost function.

**Figure 13:** Validation loss analysis on Dataset-1 and Dataset-2 over 50 epochs.

**Table 1:** Sensitivity, specificity, precision, *F*1-score, and accuracy values of different frameworks.

Method	Performance metrics				
	Sensitivity	Specificity	Precision	*F*1-score	Accuracy
Nonhierarchical structure	0.9137	0.9267	0.9384	0.9259	0.9267
The proposed method	0.9900	1.0000	1.0000	0.9950	0.9967

**Table 2:** Sensitivity, specificity, precision, *F*1-score, and accuracy values of different models.

Method	Performance metrics				
	Sensitivity	Specificity	Precision	*F*1-score	Accuracy
Single ResNet	0.9289	0.9365	0.9497	0.9348	0.9351
Single DenseNet	0.8990	0.9453	0.8900	0.8945	0.9300
The proposed method	0.9900	1.0000	1.0000	0.9950	0.9967

**Table 3:** Results using different classification models for COVID-19 detection.

Method	Performance metrics				
	Sensitivity	Specificity	Precision	*F*1-score	Accuracy
DenseNet-121 [19]	0.9159	0.9200	0.9227	0.9193	0.9200
Chen et al. [30]	0.9693	0.9700	0.9707	0.9701	0.9700
VGG-16 [14]	0.8724	0.8900	0.9133	0.8924	0.8900
Xception [35]	0.6800	0.6800	0.9273	0.7846	0.6800
Apostolopoulos et al. [31]	0.9487	0.9533	0.9604	0.9545	0.9533
Gayathri et al. [22]	0.9754	0.9402	0.9435	0.9596	0.9583
Bargshady et al. [13]	0.9001	0.8755	0.8877	0.8990	0.8769
Irfan et al. [32]	0.8824	0.9222	0.5945	0.7112	0.9220
Almalki et al. [33]	0.9628	0.9621	0.9628	0.9628	0.9625
Nguyen et al. [34]	0.9628	0.9633	0.9638	0.9633	0.9633
DualCheXNet [23]	0.8051	0.8100	0.9959	0.8904	0.8100
The proposed method	0.9900	1.0000	1.0000	0.9950	0.9967

## Data Availability

The dataset is available on the website: https://www.kaggle.com/tawsifurrahman/covid19-radiography-database/.
